# The Effect of MCM3AP-AS1/miR-211/KLF5/AGGF1 Axis Regulating Glioblastoma Angiogenesis

**DOI:** 10.3389/fnmol.2017.00437

**Published:** 2018-01-09

**Authors:** Chunqing Yang, Jian Zheng, Yixue Xue, Hai Yu, Xiaobai Liu, Jun Ma, Libo Liu, Ping Wang, Zhen Li, Heng Cai, Yunhui Liu

**Affiliations:** ^1^Department of Neurosurgery, Shengjing Hospital of China Medical University, Shenyang, China; ^2^Liaoning Research Center for Clinical Medicine in Nervous System Disease, Shenyang, China; ^3^Key Laboratory of Neuro-oncology in Liaoning Province, Shenyang, China; ^4^Department of Neurobiology, College of Basic Medicine, China Medical University, Shenyang, China; ^5^Key Laboratory of Cell Biology, Ministry of Public Health of China, and Key Laboratory of Medical Cell Biology, Ministry of Education of China, Shenyang, China

**Keywords:** angiogenesis, glioblastoma, MCM3AP-AS1, miR-211, KLF5, AGGF1

## Abstract

Glioblastoma (GBM) is the most aggressive and malignant primary tumor. Angiogenesis plays a critical role in the progression of GBM. Previous studies have indicated that long non-coding RNAs (lncRNAs) are abnormally expressed in various cancers and participate in the regulation of the malignant behaviors of tumors. The present study demonstrated that lncRNA antisense 1 to Micro-chromosome maintenance protein 3-associated protein (MCM3AP-AS1) was upregulated whereas miR-211 was downregulated in glioma-associated endothelial cells (GECs). Knockdown of MCM3AP-AS1 suppressed the cell viability, migration, and tube formation of GECs and played a role in inhibiting angiogenesis of GBM *in vitro*. Furthermore, knockdown of MCM3AP-AS1 increased the expression of miR-211. Luciferase reporter assay implicated that miR-211 targeted KLF5 3′-UTR and consequently inhibited KLF5 expression. Besides, in this study we found that MCM3AP-AS1 knockdown decreased KLF5 and AGGF1 expression by upregulating miR-211. In addition, KLF5 was associated with the promoter region of AGGF1. Knockdown of KLF5 decreased AGGF1 expression by transcriptional repression, and also inhibited the activation of PI3K/AKT and ERK1/2 signaling pathways. Overall, this study reveals that MCM3AP-AS1/miR-211/KLF5/AGGF1 axis plays a prominent role in the regulation of GBM angiogenesis and also serves as new therapeutic target for the anti-angiogenic therapy of glioma.

## Introduction

Glioblastoma (GBM) is considered to be the most common and malignant primary tumor with high aggressiveness and poor prognosis in human central nervous system (Popescu et al., 2014). One of the most prominent features of GBM is the *de novo* generation of new blood vessels. Meanwhile, as an angiogenic solid tumor, the progression of GBM depends on the nourishment of blood vessels (Jovcevska et al., 2013; Zinnhardt et al., 2017). Although surgical resection, radiotherapy, and chemotherapy have made great progress in GBM treatment in recent years (Cruceru et al., 2013), GBM patients who received comprehensive multi-mode treatment bear the median survival time of only 15 months (Codrici et al., 2016). Lately, as a brand new therapeutic strategy, the anti-angiogenic therapy has presented a deep involvement in GBM treatment (Wick et al., 2016).

Angiogenesis, characterized by the formation of new blood vessels from the existing vessels (Betz et al., 2016), plays a pivotal role in the malignancy, development, and progression of GBM. A variety of angiogenic factors are involved in the regulation of GBM angiogenesis by modulating glioma-associated endothelial cells (GECs). Furthermore, the biological behaviors of GECs, which is closely linked with GBM microenvironment, is responsible for the GBM angiogenesis (Hosono et al., 2017; Oh et al., 2017).

Long non-coding RNAs (lncRNAs), a kind of non-coding RNAs which are more than 200 nucleotides without protein coding function, have been proven to play critical roles in the regulation of cellular biological behaviors such as cell proliferation, differentiation, imprint regulation and immune response (Johnsson et al., 2014). Deregulated lncRNAs are closely related to the development and progression of malignant tumors. For example, lncRNA-MALAT1 functions as an oncogene in hepatocellular carcinoma (Malakar et al., 2017), while lncRNA-MEG3 plays a tumor suppressive role in functional pancreatic neuroendocrine tumor (Iyer et al., 2017). Micro-chromosome maintenance protein 3 (MCM3) is a vital regulator in DNA replication. MCM3AP is acetylated MCM3 with the combination of chromatin. Overexpression of MCM3AP inhibits DNA replication via the blockage of the S phase of cell cycle. The inhibition of cell proliferation mainly depends on the activity of MCM3AP acetylase (Poole et al., 2012). MCM3AP gene is located in human chromosome 21. MCM3AP participates in the regulation of gene expression in various human malignant tumors, and plays different regulatory roles (Kuwahara et al., 2016). For instance, it has been proven that MCM3AP is lowly expressed in breast carcinoma, glioma as well as other solid tumors and functions as a tumor suppressor (Ohta et al., 2009; Kuwahara et al., 2016). On the contrary, MCM3AP is highly expressed in B-cell lymphoma and hematological malignancy and acts as an oncogene (Singh et al., 2013; Kuwahara et al., 2016). MCM3AP-AS1 is a lncRNA antisense to human MCM3AP gene. The expression level of MCM3-AP1 in GECs and its potential function in GECs-dependent GBM angiogenesis remain unclear.

miRNAs are highly conserved small non-coding RNAs containing about 20 nucleotides. It is well-established that miRNAs directly target and bind to mRNAs, which in turn negatively regulate the expression of target genes (Tsikrika et al., 2017). miR-211 is located in intron 6 of the TRPM1 gene on chromosome 15 (Margue et al., 2013). A recent publication has shown that miR-211 exerts tumor suppressive function in colorectal cancer through inhibiting the proliferation, migration, and invasion of colorectal cancer cells (Sumbul et al., 2015). Moreover, it has been reported that expression of miR-211 is downregulated in glioma tissues. Overexpression of miR-211 inhibits cell proliferation and promotes cell apoptosis in U87, U4910, and U4302 glioma cell lines (Asuthkar et al., 2012; Zhang J. et al., 2017). However, the effect of miR-211 on GBM angiogenesis is still obscure.

Krüppel-like factors 5 (KLF5) is a member of the KLF transcription factor families. Recent studies have shown that KLF5 is principal in regulating cell proliferation, migration, apoptosis, and angiogenesis (Marrero-Rodriguez et al., 2014). Furthermore, it has been discovered to be singularly expressed in malignant tumors. For example, KLF5 is upregulated in cervical cancer, whereas it is lowly expressed in renal clear cell carcinoma (Fu et al., 2017). It has been reported that KLF5 is highly expressed in U87 GBM cells (Sciorra et al., 2012). However, the role of KLF5 in GBM angiogenesis is not fully understood.

Aberrant expression of angiogenic factor with G-patch and FHA domain 1 (AGGF1) has been found in congenital vascular malformations such as Klippel-Trenaunay syndrome (Zhan et al., 2016). AGGF1, previously identified as a pro-angiogenic factor, is associated with the proliferation, migration, and other biological behaviors of endothelial cells (Fan et al., 2009). A recent study in hepatocellular carcinoma and gastric cancer reveals that AGGF1 is upregulated in tumor tissues and its overexpression promotes the malignant biological behaviors of hepatocellular carcinoma and gastric cancer cells. Moreover, the elevated level of AGGF1 is positively correlated with the angiogenesis of hepatocellular carcinoma and gastric cancer (Wang W. et al., 2015; Yao et al., 2017). However, the expression level of AGGF1 in GECs and its potential function in GBM angiogenesis remains uncharted.

The primary objective of this study was to investigate the expression levels of MCM3AP-AS1, miR-211, KLF5, and AGGF1 in GECs and their potential function in GBM angiogenesis. The interactions between these factors were further explored. Their regulatory effect on angiogenesis in GBM was clearly demonstrated. The ultimate goal of this study was to establish a new basis for the anti-angiogenic and targeted molecular therapy of glioma.

## Materials and Methods

### Cell Culture

The immortalized human brain EC line hCMEC/D3 was obtained from Dr. Couraud (Institut Cochin, Paris, France). ECs were cultured as previously described (Ma et al., 2014). ECs were limited with the passage below 35. Human GBM cell line U87 and human embryonic kidney 293T (HEK293T) cells were acquired from Shanghai Institutes for Biological Sciences Cells Resource Center. They were cultured in high glucose Dulbecco’s Modified Eagle Medium (DMEM) supplemented with 10% fetal bovine serum (FBS, Gibco, Carlsbad, CA, United States). Glioma conditioned medium was obtained from the human GBM cell line U87 as previously described (Cai et al., 2015). U87 cells were plated in 100-mm-diameter Petri dishes. When they were at 70–80% confluence, we washed the incubator twice with serum free medium and then incubated the cells at the condition of 37°C with 5% CO_2_ for 24 h in serum free EBM-2 medium in a humidified incubator. Then we collected solution, centrifuged it at 800*g* at 4°C for 5 min and harvested the supernatant. Finally, we replenished it with 5% FBS, 1% penicillin-streptomycin, 1% chemically defined lipid concentrate, 1 ng/ml bFGF, 1.4 μM hydrocortisone, 5 μg/ml ascorbic acid,10 mM HEPES, EGF and hydrocortisone and stored it at 4°C. The Glioma conditioned medium, was used to culture the endothelial cells for 24 h in order to produce the GECs. All cells were maintained in a humidified incubator at 37°C with 5% CO_2_.

### Quantitative Real-time PCR

TRIzol reagent (Life Technologies Corporation, Carlsbad, CA, United States) was used to extract total RNA from ECs and GECs. RNA concentration and quality of each sample were determined with Nanodrop Spectrophotometer (ND-100) by the 260/280 nm ratio. The primers for MCM3AP-AS1, KLF5, and GAPDH were synthesized from Takara Bio (Japan). The primers for miR-211 and U6 were synthesized from the Applied Biosystems. The expression levels of MCM3AP-AS1, KLF5, and GAPDH were measured with One-Step SYBR PrimeScript RT-PCR Kit (Perfect Real Time; Takara Bio, Inc., Japan). MCM3AP-AS1: forward 5′-GCTGCTAATGGCAACACTGA-3′, reverse 5′-AGGTGCTGTCTGGTGGAGAT-3′; KLF5: forward 5′-GAACGTCTTCCTCCCTGACA-3′, reverse 5′-GGCAGTCGTTTCACTCTGGT-3′. MCM3AP: forward 5′-TGGGATTCAGACGCTTTCGC-3′, reverse 5′-TCCACAGCATCAATGGCACC-3′; TRPM1: forward 5′-GCAAACAGGTGGAGACTCAGC-3′, reverse 5′-ATTGGAATATCCGCCACCCTG-3′; GAPDH: forward 5′-CAGGAGGCATTGCTGATGAT-3′, reverse 5′-GAAGGCTGGGGCTCATTT-3′. The expression levels of miR-211 and U6 (Applied Biosystems, Foster City, CA, United States) were examined with High Capacity cDNA Reverse Transcription Kits (Applied Biosystems, Foster City, CA, United States) and Taqman Universal Master Mix II (Life Technologies Corporation, Carlsbad, CA, United States). The relative quantification 2^-ΔΔCt^ method was applied to calculate the gene expression.

### Cell Transfection

Four short-hairpin MCM3AP-AS1 (sh-MCM3AP-AS1) plasmids and the respective non-targeting sequences (negative control, NC) (sh-NC) were synthesized (Geenseed Biotech Co., Guangzhou, China). KLF5 full length (with 3′-UTR) (KLF5(+) or KLF5) plasmid, short-hairpin KLF5 (sh-KLF5) plasmid, KLF5 (without 3′-UTR) (KLF5 (non-3′UTR)) plasmid and their respective non-targeting sequences (negative control, NC) (KLF5-NC or sh-NC), short-hairpin AGGF1 (sh-AGGF1) plasmid and the respective non-targeting sequences (negative control, NC) (sh-NC) were constructed (Life Technologies, Waltham, MA, United States). After seeded into 24-well plates (Corning), ECs were transfected with the plasmids via LTX and Plus reagent (Life Technologies) when they were at 70–80% confluence. Geneticin (G418; Sigma–Aldrich, St. Louis, MO, United States) was utilized to select the G418-resistant clones after 3∼4 weeks. miR-211 agomir (miR-211(+)), miR-211 antagomir (miR-211(-)) and their respective non-targeting sequences (negative control, NC) (miR-211(+)-NC or miR-211(-)-NC) (GenePharma, Shanghai, China) were transiently transfected into ECs using Opti-MEM and Lipofectamine 3000 reagent (Life Technologies Corporation, Carlsbad, CA, United States) when the confluence reached 70∼80%. Cells were collected at 48 h after transfection.

### Cell Proliferation Assay

Cell Counting Kit-8 (CCK-8, Beyotime Institute of Biotechnology, Jiangsu, China) assay was conducted for the cell proliferation assay. Cells were plated in 96-well plates at the density of 2000 cells per well, then added with 10 μL of the CCK-8 solution. Cells were incubated in a humidified incubator at 37°C for 2 h. The absorbance at 450 nm was measured with the SpectraMax M5 microplate reader (Molecular Devices, United States).

### Cell Migration Assay

The upper chamber of a 24-well transwell chamber (8 μm pore size, Corning Inc., Corning, NY, United States) was used to incubate the cells resuspended in 200 μL serum-free medium at a density of 2 × 10^5^∼4 × 10^5^ cells per ml, and 600 μL of the EBM-2 medium supplemented with 5% FBS was added to the lower chamber. After incubation at 37°for 48 h, the cells on the upper membrane surface were removed. Cells on the lower surface of the membrane were fixed with methanol and glacial acetic acid at the ratio of 3:1 and stained with 10% Giemsa (Dinguo, China). Then five randomly selected fields were counted for statistical analysis in each well.

### Tube Formation Assay

The 96-well plates were coated with 100 μL Matrigel (BD Biosciences, Bedford, MA, United States) per well and maintained at 37°C for 30 min. Then the cells were added to Matrigel-coated wells which were resuspended in 100 μL complete EBM-2 medium at the concentration of 4 × 10^5^/mL and incubated at 37°C for 24 h. Olympus DP71 immunofluorescence microscopy (Olympus, Tokyo, Japan) was applied to collect the photos and the Chemi Imager 5500 V2.03 software (Alpha Innotech, San Leandro, CA, United States) was used to measure the total tubule length and numbers of tubule branches.

### Western Blot Analysis

Total proteins from the cells on ice were extracted by RIPA buffer with protease inhibitors (Beyotime Institute of Biotechnology). Electrophoresis was conducted to equal amount of protein samples (40 μg) with sodium dodecyl sulfate–polyacrylamide gel electrophoresis (SDS–PAGE) and then transferred to PVDF membranes. Membranes were incubated in 5% non-fat milk dissolved in Tris-buffered saline (TBS) containing 0.1% Tween-20 for 2 h at room temperature and then incubated with primary antibodies against KLF5 (1:500, Santa Cruz Biotechnology), AGGF1 (1:2000, Proteintech, Chicago, IL, United States), p-PI3K (1:500, Bioworld, Minneapolis, MN, United States), PI3K (1:1,000, CST, EUGENE), p-AKT (1:2,000, CST, EUGENE), AKT (1:2,000, CST, EUGENE), p-ERK1/2 (1:1,000, CST, EUGENE), ERK1/2 (1:1,000, CST, EUGENE), MCM3AP (1:500, Proteintech, Chicago, IL, United States), and GAPDH (1:1000, Proteintech, Chicago, IL, United States) at 4°C overnight. On next day, membranes were incubated with secondary antibodies (goat anti-rabbit or goat anti-mouse, 1:5000, respectively; Santa Cruz Biotechnology, Santa Cruz, CA, United States) at room temperature for 2 h. Immunoblots were visualized by enhanced chemiluminescence (ECL kit, Santa Cruz Biotechnology) and scanned using ChemImager 5,500 V2.03 software. Then FluorChem 2.0 software was used to calculate the integrated density values (IDV).

### Reporter Vectors Construction and Luciferase Reporter Assays

The potential binding sites of miR-211 in MCM3AP-AS1 and KLF5 3′-UTR sequences were amplified by PCR and cloned into a pmirGlo Dual-luciferase miRNA Target Expression Vector (Promega, Madison, WI, United States) to construct luciferase reporter vector (MCM3AP-AS1-Wt and KLF5-Wt, GenePharma). The sequence of putative binding site was replaced as indicated (MCM3AP-AS1-Mut and KLF5-Mut) to mutate the putative binding site of MCM3AP-AS1 or KLF5. HEK-293T cells were seeded in 96-well plates and were co-transfected with MCM3AP-AS1-Wt (or MCM3AP-AS1-Mut) or KLF5-Wt (or KLF5-Mut) and miR-211 or miR-211-NC plasmids when the confluence reached at 70∼80%. Dual-Luciferase reporter assay kit (Promega) was then applied to measure the luciferase activities at 48 h after the transfection. The cells were divided into five groups, respectively: Control group, MCM3AP-AS1-Wt+miR-211-NC group (transfected with MCM3AP-AS1-Wt and miR-211-NC), MCM3AP-AS1-Wt+miR-211 group (transfected with MCM3AP-AS1-Wt and miR-211), MCM3AP-AS1-Mut+miR-211-NC group (transfected with MCM3AP-AS1-Mut and miR-211-NC), MCM3AP-AS1-Mut+miR-211 group (transfected with MCM3AP-AS1-Mut and miR-211); Control group, KLF5-Wt+miR-211-NC group (transfected with KLF5-Wt and miR-211-NC), KLF5-Wt+miR-211 group (transfected with KLF5-Wt and miR-211), KLF5-Mut+miR-217-NC group (transfected with KLF5-Mut and miR-211-NC), KLF5-Mut+miR-211 group (transfected with KLF5-Mut and miR-211).

### Chromatin Immunoprecipitation Assay (ChIP)

Simple ChIP Enzymatic Chromatin IP Kit (Cell Signaling Technology, Danvers, MA, United States) was used for ChIP assays according to the manufacturer’s instructions. Briefly, cells were crosslinked with EBM-2 containing 1% formaldehyde and collected in lysis buffer. Then the chromatin was digested by micrococcal nuclease. Immunoprecipitation was incubated with 3 μg of anti-KLF5 antibody (Santa Cruz Biotechnology) or normal rabbit IgG followed by immunoprecipitating with Protein G Agarose Beads and stored at 4°C overnight with gentle shaking. Then the DNA crosslink was reversed by 5 mol/L NaCl and Proteinase K and finally DNA was purified. Immunoprecipitated DNAs were amplified by PCR according to their specific primers as follows: Control PCR1: forward 5′-AGCACCTTAATGCAATTCCTGA-3′, reverse 5′-GCAGTGCTCCTCTTATTTGTCT-3′; AGGF1 PCR2: forward 5′-CGCTCTTAGGGCTTCGGTAG-3′, reverse 5′-GAAAGCGGGAAGACCTGACA-3′.

### *In Vivo* Matrigel Plug Assay

Matrigel plug assay was conducted to measure the angiogenesis as previously described (Jia et al., 2016). Nude mice were purchased from the Vital River Laboratory Animal Technology Co., Ltd. (Beijing, China). All the male BALB/c athymic nude mice were fed with autoclaved food and water during the experiment. All the experiments with nude mice were performed strictly in accordance with the protocol approved by the Administrative Panel on Laboratory Animal Care of Shengjing Hospital.

In brief, GECs resuspended in 400 μL of solution containing 80% Matrigel at a density of 3 × 10^5^ cells per ml were subcutaneously injected. Plugs were obtained after 4 days and then weighed, photographed, and dispersed in 400 μL of PBS (overnight incubation at 4°C) to collect the hemoglobin. Hemoglobin content was measured using Drabkin’s solution (Sigma) according to manufacturer’s instructions.

### Statistical Analysis

Quantitative data were presented as mean ± standard deviation (SD). SPSS 18.0 statistical software was applied with the Student’s *t*-test or one-way analysis of variance ANOVA to evaluate all statistical analyses. Differences were considered to be statistically significant when *P* < 0.05.

## Results

### Knockdown of MCM3AP-AS1 Inhibits the Angiogenesis of GECs

Quantitative real-time PCR was conducted to evaluate the endogenous expression of MCM3AP-AS1 in GECs and ECs. As shown in **Figure 1A**, the expression of MCM3AP-AS1 was significantly increased in GECs compared with that in ECs (*P* < 0.01). Then we demonstrated the impact of MCM3AP-AS1 knockdown on the process of cell viability, migration and tube formation in GECs. As shown in **Figure 1B**, the viability of GECs was decreased in sh-MCM3AP-AS1 group compared with sh-NC group (*P* < 0.05). Further, transwell migration assays were used to verify the migration ability of GECs. The results showed that the number of migrated cells was decreased in sh-MCM3AP-AS1 group compared with that in sh-NC group (*P* < 0.05) in **Figure 1C**. **Figure 1D** demonstrated the results of tube formation assay. Relative tubule length and number of branches were decreased in sh-MCM3AP-AS1 group compared with sh-NC group (*P* < 0.05). Meanwhile, **Figures 1E,F** illustrated that KLF5 mRNA and protein level expression were both robustly decreased in GECs (*P* < 0.01). The western blot assays showed that the expression of KLF5 and AGGF1 were significantly decreased in sh-MCM3AP-AS1 group compared with that in sh-NC group (*P* < 0.01) in **Figures 1G,H**.

**FIGURE 1:** MCM3AP-AS1 expression in glioma-associated endothelial cells (GECs) and inhibition of MCM3AP-AS1 knockdown on glioblastoma (GBM) angiogenesis, KLF5, and AGGF1 expression. **(A)** Relative MCM3AP-AS1 expression in ECs and GECs by quantitative real-time PCR. Data are presented as mean ± SD. (*n* = 5, each group), *^∗^P <* 0.01 vs. ECs group. **(B)** CCK-8 assay was used to evaluate the effect of MCM3AP-AS1 knockdown on GECs proliferation. **(C)** Effect of MCM3AP-AS1 knockdown on quantification number of GECs migration. **(D)** Effect of MCM3AP-AS1 knockdown on GECs tube formation. Data are presented as mean ± SD. (*n* = 5, each group), *^∗^P <* 0.05 vs. sh-NC group. **(E)** Relative KLF5 mRNA expression in ECs and GECs by quantitative real-time PCR. **(F)** Relative KLF5 expression in ECs and GECs by Western blot assay. **(G)** The effect of MCM3AP-AS1 knockdown on expression of KLF5 by Western blot assay. **(H)** The effect of MCM3AP-AS1 knockdown on expression of AGGF1. Data are presented as mean ± SD. (*n* = 5, each group), *^∗^P <* 0.01 vs. sh-NC group. Scale bars represent 30 μm.

### Overexpression of miR-211 Inhibits the Angiogenesis of GECs

**Figure 2A** shows that the expression of miR-211 is significantly decreased in GECs compared with that in ECs (*P* < 0.01) using qRT-PCR. Meanwhile, we also evaluated the expression level of TRPM1 mRNA which was also decreased in GECs compared with that in ECs (Supplementary Figure 1A; *P* < 0.01). In addition, as shown in Supplementary Figure 1B, miR-211 and TRPM1 mRNA expression were both upregulated in pre-miR-211 group compared with pre-NC group (*P* < 0.01). Subsequently, we verified the expression of KLF5 mRNA and KLF5 protein level as we upregulated or downregulated miR-211 in GECs. These results demonstrated that there was no difference of the KLF5 mRNA level in pre-miR-211 group and anti-miR-211 group (**Figure 2B**; *P* > 0.05) while the expression of KLF5 protein level was downregulated in pre-miR-211 group (**Figure 2C**; *P* < 0.01). On the contrary, it was upregulated in anti-miR-211 group (*P* < 0.01). As shown in **Figures 2D–F**, the upregulation of miR-211 inhibited the cell viability, migration, and tube formation of GECs in pre-miR-211 group compared with pre-NC group (*P* < 0.05), whereas the downregulation of miR-211 promoted the cell viability, migration, and tube formation of GECs in anti-miR-211 group compared with anti-NC group (*P* < 0.05). **Figure 2G** shows the results of the western blot assays that AGGF1 protein level is downregulated in pre-miR-211 group (*P* < 0.01), while it is upregulated in anti-miR-211 group (*P* < 0.01).

**FIGURE 2:** miR-211 expression in GECs and regulation of miR-211 on GBM angiogenesis, KLF5 and AGGF1 expression. **(A)** Relative miR-211 expression in ECs and GECs by quantitative real-time PCR. Data are presented as mean ± SD. (*n* = 5, each group), *^∗^P <* 0.01 vs. ECs group. **(B,C)** Effect of miR-211 on the expression of KLF5 mRNA and KLF5 protein level. **(D)** CCK-8 assay was used to evaluate the effect of miR-211 on GECs proliferation. **(E)** Effect of miR-211 on quantification number of GECs migration. **(F)** Effect of miR-211 on GECs tube formation. Data are presented as mean ± SD. (*n* = 5, each group), *^∗^P <* 0.05 vs. pre-NC group; *^#^P <* 0.05 vs. anti-NC group. **(G)** The effect of miR-211 on expression of AGGF1 by Western blot assay. Data are presented as mean ± SD. (*n* = 5, each group), *^∗^P <* 0.01 vs. pre-NC group; *^#^P <* 0.01 vs. anti-NC group. Scale bars represent 30 μm.

### miR-211 Targets MCM3AP-AS1 in GECs

We first detected the expression of miR-211 in GECs with MCM3AP-AS1 inhibition. As shown in **Figure 3A**, miR-211 expression was increased in sh-MCM3AP-AS1 group compared with sh-NC group (*P* < 0.01). Moreover, **Figure 3A** also shows that MCM3AP-AS1 expression is negatively correlated with miR-211 expression in GECs (*P* < 0.01). In the meantime, Supplementary Figure 1C shows that TRPM1 mRNA expression has the same trend with miR-211 expression in sh-MCM3AP-AS1 group. Then bioinformatics database (Starbase) suggested that there was a putative binding site between MCM3AP-AS1 and miR-211. **Figure 3B** shows the results of the dual-luciferase reporter assay which confirmed the binding site between MCM3AP-AS1 and miR-211. Meanwhile, luciferase activity was significantly reduced in MCM3AP-AS1-Wt + miR-211 group compared with MCM3AP-AS1-Wt + miR-211-NC group (*P* < 0.05). **Figure 3B** substantiated that miR-211 targeted MCM3AP-AS1 by the functional binding site. Furthermore, RNA-binding protein immunoprecipitation (RIP) experiment was performed to determine whether MCM3AP-AS1 and miR-211 were in a RNA-induced silencing complex (RISC). **Figure 3C** shows MCM3AP-AS1 and miR-211 are both enriched in anti-Ago2 group (*P* < 0.01). These results indicated the mechanism where MCM3AP-AS1 negatively regulated miR-211 expression in a RISC. In addition, the expression levels of MCM3AP mRNA and MCM3AP protein were both increased in sh-MCM3AP-AS1 group and also in pre-miR-211 group (Supplementary Figures 2A,B; *P* < 0.01). Supplementary Figures 2A,B also shows that the expression levels of MCM3AP mRNA and MCM3AP protein were increased in sh-MCM3AP-AS1+pre-miR-211 group while silencing miR-211 can reverse this effect (*P* < 0.01). Further, **Figures 3D–F** shows that the cell viability, migration, and tube formation of GECs associated with the down-regulation of MCM3AP-AS1 is reversed by silencing miR-211. In addition, **Figures 3G,H** shows the KLF5 and AGGF1 protein expression levels are significantly decreased in sh-MCM3AP-AS1+pre-miR-211 group, while silencing miR-211 reversed the effect of down-regulation of MCM3AP-AS1 on KLF5 and AGGF1 protein expression (*P* < 0.01).

**FIGURE 3:** Knockdown of MCM3AP-AS1 inhibited GBM angiogenesis, KLF5 and AGGF1 expression via increasing miR-211 expression. **(A)** Quantitative real-time PCR analysis for miR-211 expression negatively correlative with MCM3AP-AS1 in GECs. Data are presented as mean ± SD. (*n* = 5, each group), *^∗^P <* 0.01 vs. sh-NC group, *^∗^P <* 0.01 vs. pre-NC group; *^#^P <* 0.01 vs. anti-NC group. **(B)** The predicted miR-211 binding site in MCM3AP-AS1 and the designed mutant sequences. Dual-luciferase report assay of HEK293T cells co-transfected with MCM3AP-AS1-Wt and miR-211-NC or MCM3AP-AS1-Wt and miR-211, and MCM3AP-AS1-Mut and miR-211-NC or MCM3AP-AS1-Mut and miR-211. Data are presented as mean ± SD. (*n* = 5, each group), *^∗^P <* 0.05 vs. MCM3AP-AS1-Wt + miR-211-NC group. **(C)** miR-211 was identified in MCM3AP-AS1-RISC complex. Relative expression levels of MCM3AP-AS1 and miR-211 were determined by quantitative real-time PCR. Data are presented as mean ± SD. (*n* = 5, each group), *^∗∗^P* < 0.01 vs. anti-normal IgG group. **(D)** CCK-8 assay was conducted to evaluate the effect of MCM3AP-AS1 and miR-211 on GECs proliferation. **(E)** Effect of MCM3AP-AS1 and miR-211 on quantification number of GECs migration. **(F)** Effect of MCM3AP-AS1 and miR-211 on GECs tube formation. Data are presented as mean ± SD. (*n* = 5, each group). *^∗^P <* 0.05 vs. sh-NC + pre-NC group. **(G)** The effect of MCM3AP-AS1 and miR-211 on expression of KLF5 by Western blot assay. **(H)** The effect of MCM3AP-AS1 and miR-211 on expression of AGGF1 by Western blot assay. Data are presented as mean ± SD. (*n* = 5, each group), *^∗^P <* 0.01 vs. sh-NC + pre-NC group. Scale bars represent 30 μm.

### Knockdown of KLF5 Inhibits the Biological Behaviors of GECs by Inhibiting the Expression of AGGF1 and the Activity of PI3K/AKT/ERK1/2 Signaling Pathways

As shown in **Figures 4A,B**, AGGF1 mRNA and protein level expression were directly decreased in KLF5 (-) group compared with KLF5 (-)-NC group (*P* < 0.01). Furthermore, cell viability, migration, and tube formation of GECs were suppressed in KLF5 (-) group which indicated that knockdown of KLF5 inhibited the process of angiogenesis in GECs (**Figures 4C–E**). In addition, we examined the expression of proteins involved in PI3K, AKT, ERK1/2 signaling pathways. The expression levels of p-PI3K, p-AKT, and p-ERK1/2 were signally decreased in KLF5 (-) group (**Figure 4F**; *P* < 0.05). We further utilized JASPA database to propose there was a binding set between KLF5 and AGGF1 protein, and we predicted the promoter sequence of AGGF1 and transcription start sites (TSSs) at the same time. Then we identified the potential binding site by scanning the DNA sequence from 1000 bp region upstream and 200 bp region downstream of TSS. Simultaneously, as shown in **Figure 4G**, KLF5 directly bound to the promoter region of AGGF1 in GECs, while in the corresponding negative control group, there was no combination between KLF5 and the control region. The above results demonstrated there was a direct association between KLF5 and the promoter sequence of AGGF1 in GECs.

**FIGURE 4:** KLF5 exerted oncogenic role and could modulate AGGF1 expression by binding to its promoter region in GECs. **(A,B)** Effect of KLF5 knockdown on the expression of AGGF1 mRNA and AGGF1 protein level. **(C)** CCK-8 assay was applied to evaluate the effect of KLF5 knockdown on GECs proliferation. **(D)** Effect of KLF5 knockdown on quantification number of GECs migration. **(E)** Effect of KLF5 knockdown on GECs tube formation. Data are presented as mean ± SD. **(F)** Western blot analysis of p-PI3K, PI3K, p-AKT, AKT, p-ERK1/2, and ERK1/2 regulated by KLF5 in GECs, using GAPDH as endogenous control. Data are presented as mean ± SD. (*n* = 5, each group), *^∗^P <* 0.05 vs. KLF5 (-)-NC group. **(G)** KLF5 bound to the promoter region of AGGF1 in GECs. Putative KLF5 binding sites are indicated. Immunoprecipitated DNA was amplified by PCR. Normal rabbit IgG was used as a negative control. Scale bars represent 30 μm.

### KLF5 Is a Target of miR-211

According to the bioinformatics database (miRanda), KLF5 was identified as a target of miR-211. Dual-luciferase reporter assay was performed to confirm the above mentioned binding site. As shown in **Figure 5A**, the luciferase activity in the KLF5-Wt+miR-211 group was significantly decreased compared with KLF5-Wt+miR-211-NC group (*P* < 0.05). The results indicated that KLF5 combined with miR-211 and acted as a target of miR-211. The following results confirmed that KLF5 rescued miR-211-induced impact of malignant progression of GECs. We established GECs stably expressing miR-211+KLF5 (non-3′UTR) and then detected the angiogenesis. As shown in **Figures 5B–D**, the cell viability, migration, and tube formation of GECs in miR-211+KLF5 (non-3′UTR) group were markedly restored compared with that in miR-211+KLF5 group (*P* < 0.05). Furthermore, we demonstrated that p-PI3K, p-AKT, and p-ERK1/2 levels were prominently increased in miR-211+KLF5 (non-3′UTR) group compared with miR-211+KLF5 group (**Figures 5E,F**; *P* < 0.01).

**FIGURE 5:** miR-211 inhibited GBM angiogenesis via regulating PI3K/AKT and ERK1/2 pathways by targeting to KLF5 3′-UTR. **(A)** The predicted miR-211 binding site in KLF5 and the designed mutant sequences were indicated. Dual-luciferase report assay of HEK 293T cells co-transfected with KLF5-Wt and miR-211-NC or KLF5-Wt and miR-211, and KLF5-Mut and miR-211-NC or KLF5-Mut and miR-211. Data are presented as mean ± SD. (*n* = 5, each group), *^∗^P <* 0.05 vs. KLF5-Wt + miR-211-NC group. **(B)** CCK-8 assay was performed to evaluate the effect of miR-211 and KLF5 on GECs proliferation. **(C)** Effect of miR-211 and KLF5 on quantification number of GECs migration. **(D)** Effect of miR-211 and KLF5 on GECs tube formation. Data are presented as mean ± SD. (*n* = 5, each group), *^∗^P <* 0.05 vs. miR-211+KLF5 group; *^#^P <* 0.05 vs. miR-211+KLF5-NC group. **(E)** The effect of miR-211 and KLF5 on expression of AGGF1 by Western blot assay. **(F)** Western blot analysis of p-PI3K, PI3K, p-AKT, AKT, p-ERK1/2, and ERK1/2 regulated by miR-211 and KLF5 in GECs, shown using GAPDH as endogenous control. Data are presented as mean ± SD. (*n* = 5, each group), *^∗^P <* 0.01 vs. miR-211+KLF5 group; *^#^P <* 0.01 vs. miR-211+KLF5-NC group. Scale bars represent 30 μm.

### Knockdown of AGGF1 Inhibits the Angiogenesis of GECs

**Figures 6A,B** demonstrated that AGGF1 mRNA and protein level were both significantly upregulated in GECs (*P* < 0.01). As shown in **Figure 6C**, we used CCK-8 assays to detect the viability of GECs. Cell viability was decreased in AGGF1 (-) group compared with AGGF1 (-)-NC group (*P* < 0.05). Also, transwell migration assays were conducted to verify the migration ability of GECs. The number of migrating cells was decreased in AGGF1 (-) group compared with that in AGGF1 (-)-NC group (**Figure 6D**; *P* < 0.05). As shown in **Figure 6E**, the results of tube formation assay revealed relative tubule length and number of branches were significantly decreased in AGGF1 (-) group compared with that in the AGGF1 (-)-NC group (*P* < 0.05).

**FIGURE 6:** AGGF1 mRNA expression in GECs and inhibition of AGGF1 knockdown on proliferation, migration, and tube formation of GECs. **(A)** Relative AGGF1 mRNA expression in ECs and GECs by quantitative real-time PCR. **(B)** Relative AGGF1 expression in ECs and GECs by Western blot assay. Data are presented as mean ± SD. (*n* = 5, each group), *^∗^P <* 0.01 vs. ECs group. **(C)** CCK-8 assay was conducted to evaluate the effect of AGGF1 knockdown on GECs proliferation. **(D)** Effect of AGGF1 knockdown on quantification number of GECs migration. **(E)** Effect of AGGF1 knockdown on GECs tube formation. Data are presented as mean ± SD. (*n* = 5, each group), *^∗^P <* 0.05 vs. AGGF1 (-)-NC group. Scale bars represent 30 μm.

### Knockdown of MCM3AP-AS1, Overexpression of miR-211, and Their Combined Application Inhibits the Angiogenesis of GECs *in Vivo*

We further used Matrigel plug assay to measure the angiogenesis of GECs *in vivo*. As shown in **Figures 7A,B**, the results demonstrated that the amount of hemoglobin in sh-MCM3AP-AS1 group, pre-miR-211 group, and sh-MCM3AP-AS1+pre-miR-211 group were significantly decreased compared with Control group (*P* < 0.05). In the meantime, the amount of hemoglobin in sh-MCM3AP-AS1+pre-miR-211 group was significantly decreased compared with both sh-MCM3AP-AS1 group and pre-miR-211 group, respectively. The above results revealed that the combination of MCM3AP-AS1 knockdown and miR-211 overexpression presented the strongest inhibitory effect on GBM angiogenesis *in vivo*.

**FIGURE 7:** MCM3AP-AS1 knockdown combined with miR-211 overexpression inhibited GBM angiogenesis. **(A)** Matrigel plug assay was used to measure GBM angiogenesis. **(B)** The amount of hemoglobin was measured. Data are presented as mean ± SD. (*n* = 5, each group), *^∗^P <* 0.05 vs. Control group; *^#^P <* 0.05 vs. sh-MCM3AP-AS1 group. ^&^*P <* 0.05 vs. pre-miR-211 group.

## Discussion

In this study, we demonstrated that MCM3AP-AS1 was highly expressed in GECs. Knockdown of MCM3AP-AS1 suppressed the cell viability, migration, and tube formation of GECs *in vitro*. In contrast to MCM3AP-AS1, miR-211 was significantly downregulated in GECs. Meanwhile, inhibitory effects on GECs cell viability, migration, and tube formation were observed following the overexpression of miR-211. Besides, we confirmed that miR-211 directly targeted MCM3AP-AS1 in a sequence-dependent manner and there was a reciprocal repression between MCM3AP-AS1 and miR-211. Furthermore, elevated level of KLF5 was detected in GECs. Meanwhile, we demonstrated that restoration of miR-211 downregulated KLF5 as well as inhibited GBM angiogenesis by targeting KLF5 3′-UTR. Moreover, overexpression of KLF5 promoted the expression of AGGF1 by increasing the promoter activity of AGGF1. In addition, PI3K/AKT and ERK1/2 signaling pathways were involved in MCM3AP-AS1-mediated GBM angiogenesis. Remarkably, the *in vivo* study verified that MCM3AP-AS1 inhibition combined with the miR-211 overexpression presented the most optimal inhibitory effect on GBM angiogenesis.

Our findings provided the evidence that MCM3AP-AS1 was upregulated in GECs and knockdown of MCM3AP-AS1 inhibited the cell viability, migration, and tube formation of GECs, which were the main process of endothelial cell-dependent GBM angiogenesis. The above results indicated that MCM3AP-AS1 acted as an oncogene in GECs. A previous study shows that HOXA11 expression level is markedly decreased in renal cell carcinoma (RCC), suggesting that HOXA11 exerts tumor-suppressive function in RCC (Wang et al., 2017b). On the contrary, the antisense strand of HOXA11 (HOXA11-AS1) is upregulated in breast cancer (Li W. et al., 2017), and non-small cell lung cancer (NSCLC) (Zhang Y. et al., 2017), and acts as an oncogene. In this study, our results of the expression of MCM3AP mRNA and MCM3AP protein level were both contrary to the expression of MCM3AP-AS1. As previously reported, MCM3AP is lowly expressed in glioma (Ohta et al., 2009). Hence, the underlying mechanism involved in MCM3AP-AS1 regulating GBM angiogenesis remains further investigation. Further, we found that miR-211 was lowly expressed in GECs and the expression of the host gene TRPM1 mRNA was synchronously decreased in GECs. Meanwhile, the results in our study demonstrated that there was a same change between miR-211 expression and TRPM1 mRNA expression. Several studies have reported co-expression between miRNA and the host gene. For example, miR-218-5p is located in intron 14 of the slit guidance ligand 2 (SLIT2) gene and co-expressed in the synthesis of long-chain polyunsaturated fatty acids (Zhang M. et al., 2017). Also, miR-932 and the host gene Drosophila neuroligin2 (dnlg2) were co-expressed in Drosophila head (Qian et al., 2016). In our study, the results demonstrated that miR-211 and the host gene TRPM1 were co-expressed in GECs. Moreover, miR-211 overexpression impaired GECs proliferation, migration and tube formation. It has been proven that miR-211 is downregulated in glioma samples. Ectopic expression of miR-211 inhibits glioma cell proliferation, while promotes cell apoptosis (Asuthkar et al., 2012; Zhang J. et al., 2017). Consistent with the above findings, we demonstrated that miR-211 functioned as a tumor-suppressor in GBM angiogenesis. In addition, impaired expression of miR-211 has also been detected in melanoma, thyroid tumor, and renal cancer. In melanoma, overexpression of miR-211 reduces the cell proliferation, migration, and invasion (Mazar et al., 2010, 2016). Besides, miR-211 is downregulated in thyroid tumor and overexpression of miR-211 hinders the proliferation, migration, and invasion of thyroid tumor cells (Wang et al., 2017c). Meanwhile, *in vitro* and *in vivo* studies reveal that upregulation of miR-211 suppresses the migration and invasion in renal cancer (Wang et al., 2017a).

Bioinformatics database (Starbase) manifested MCM3AP-AS1 harbored a putative binding site of miR-211. Further, luciferase reporter assay confirmed the above binding site which indicated that miR-211 directly targeted MCM3AP-AS1. In the present study, we found that knockdown of MCM3AP-AS1 increased miR-211 expression level. Conversely, overexpression of miR-211 reduced MCM3AP-AS1 expression level, indicating that there was a reciprocal repression between MCM3AP-AS1 and miR-211. RIP assay indicated that MCM3AP-AS1 and miR-211 were coupled with Ago-2 protein in a RISC complex. Knockdown of MCM3AP-AS1 combined with overexpression of miR-211 significantly inhibited the cell viability, migration, and tube formation of GECs. These findings demonstrated that knockdown of MCM3AP-AS1 impaired GBM angiogenesis via negatively regulating miR-211. Growing evidence has indicated that lncRNAs may regulate the biological behaviors of tumor cells by serving as miRNA molecular sponges (Laneve et al., 2017; Tran et al., 2017). LncRNAs acts as competing endogenous RNAs (ceRNAs), competing for miRNA binding (Conte et al., 2017). Meanwhile, according to a previous report, non-coding RNAs usually form ribonucleoprotein (RNP) complexes with their partner proteins to exert their functions and miRNAs assemble with Argonaute (Ago) family proteins into the effector complex called RISC that mediates the target gene silencing (Kobayashi and Tomari, 2016). As a result, MCM3AP-AS1 can function as a sponge to sequester and degrade miR-211. Moreover, it has been proven that lncRNA PVT1 promotes the malignant behaviors of osteosarcoma cells through negatively regulating miR-195 (Zhou et al., 2016). In addition, lncRNA PVT1 is revealed to promote pancreatic cancer cell proliferation and migration by binding and negatively regulating miR-448 (Zhao et al., 2017). Moreover, lncRNA-PNUTS inhibits the invasion and migration of NSCLC A549 cells by down-regulating miR-205 (Grelet et al., 2017). Besides, lncRNA CCAT2 has been detected to be upregulated in colon cancer cells and knockdown of lncRNA CCAT2 suppresses colon cancer cell malignancy by upregulating miRNA-145 (Yu et al., 2017). In addition, lncRNA UCA1 is highly expressed in lung cancer. Knockdown of lncRNA UCA1 restrains the proliferation, migration, and invasion of lung cancer cells, as well as arrested cell cycle, while promotes cell apoptosis (Li D. et al., 2017).

As expected, KLF5 was verified to be upregulated in GECs in the present research. Recent studies have implied the involvement of KLF5 in the regulation of tumor progression. Meanwhile, increasing evidence has shown that KLF5 plays a pivotal role in endothelial cells. KLF5 has been found highly expressed in bladder carcinoma cells and downregulation of KLF5 restrains bladder carcinoma cell-induced angiogenesis (Chen et al., 2006; Gao et al., 2015). Moreover, previous research has proven that KLF5 is upregulated in prostate cancer cells, and knockdown of KLF5 suppresses prostate cancer cell-induced angiogenesis by inhibiting AKT pathways (Xing et al., 2014; Ci et al., 2015). Bioinformatics database predicted that KLF5 had a putative binding site of miR-211. Subsequent luciferase reporter assay confirmed that miR-211 bound to the KLF5 3′-UTR. Collectively, these results indicated that miR-211 inhibited GBM angiogenesis by targeting the 3′-UTR of KLF5. MiR-211 has been proven to affect gene expression and function by targeting the 3′-UTR. For instance, miR-211 exerts inhibitory effected on gastric cancer cell proliferation and invasion by downregulating SOX4 mRNA expression (Wang C.Y. et al., 2015). In addition, miR-211 targets KCNMA1 mRNA 3′-UTR to suppress melanoma cell migration and invasion (Mazar et al., 2010). Also, downregulation of miR-211 is involved in aberrant expression of the PRAME protein by targeting the PRAME mRNA 3′-UTR in melanoma cells (Sakurai et al., 2011). In cervical cancer, miR-211 inhibits the invasion and epithelial-to-mesenchymal transition (EMT) of cancer cells by targeting MUC4 3′-UTR (Xu et al., 2017). Consistent with the above results, we demonstrated that overexpression of miR-211 suppressed GBM angiogenesis by targeting KLF5 3′-UTR.

Findings in this study showed that AGGF1 was upregulated in GECs and knockdown of AGGF1 inhibited GBM angiogenesis. It is well accepted that AGGF1, a pro-angiogenic factor, is highly expressed in cells associated with KTS such as endothelial cells and facilitates endothelial cell proliferation, migration and tube formation *in vivo* (Timur et al., 2005; Fan et al., 2009). Aberrant expression of AGGF1 has been detected in a variety of tumors in previous studies. For example, impaired AGGF1 level is detected in bladder urothelial carcinoma (Xu et al., 2014) whereas increased AGGF1 level is observed in hepatocellular carcinoma. Moreover, elevated AGGF1 level promoted tumor angiogenesis and predicted the poor prognosis of hepatocellular carcinoma patients (Wang W. et al., 2015). *In silico* analysis (JASPAR) suggested that KLF5 was associated with the promoter sequence of AGGF1. Chromatin immunoprecipitation (ChIP) assays in this study suggested that KLF5 was associated with the promoter region of AGGF1 from -65 to -103 bp relative to the TSS. Moreover, knockdown of KLF5 impaired the expression of AGGF1 and inhibited the activity of PI3K/AKT and ERK1/2 pathways and thus suppressed GBM angiogenesis. Further, our results indicated that knockdown of KLF5 significantly decreased the expression of AGGF1 by transcriptional repression. Meanwhile, impaired activity of PI3K/AKT and ERK1/2 pathways following KLF5 knockdown might be at least partially due to the inhibition of AGGF1. Previous researches have demonstrated that overexpression of AGGF1 promotes rat cardiomyocytes and mice endothelial cells angiogenesis by activating the PI3K/AKT and ERK1/2 signaling pathways after myocardial ischemia/reperfusion injury (Liu et al., 2014). In summary, knockdown of MCM3AP-AS1 combined with overexpression of miR-211 immensely reduced the expression of KLF5 and AGGF1. These results conclusively revealed that MCM3AP-AS1/miR-211/KLF5/AGGF1 axis played a vital role in the process of GBM angiogenesis. The mechanism underlying GBM angiogenesis regulated by MCM3AP-AS1/miR-211/KLF5/AGGF1 axis is schematically presented in **Figure 8**.

**FIGURE 8:** The schematic cartoon of the mechanism of MCM3AP-AS1/miR-211/KLF5/AGGF1 axis in GBM angiogenesis.

Ultimately, there was a significant decrease in the hemoglobin content in sh-MCM3AP-AS1 group, pre-miR-211 group and sh-MCM3AP-AS1+pre-miR-211 group, which suggested the significant decrease in new vessels. Moreover, MCM3AP-AS1 knockdown combined with miR-211 overexpression presented the lowest hemoglobin content and quantities of new vessels. These results revealed that knockdown of MCM3AP-AS1 combined with overexpression of miR-211 produced the strongest inhibitory effect on GBM angiogenesis *in vivo*. Considering the results mentioned above, in order to demonstrate the effects on the GBM angiogenesis, we, respectively, utilized the inhibitor of MCM3AP-AS1 and the agonist of miR-211, or their combination as potential therapeutic agents. According to the research results we could firmly prove that there was a suppressive effect on GBM angiogenesis by these therapeutic agents.

## Conclusion

Our study demonstrated for the first time that MCM3AP-AS1, miR-211, KLF5, and AGGF1 were deregulated in GECs. Meanwhile, *in vitro* and *in vivo* studies revealed that MCM3AP-AS1/miR-211/KLF5/AGGF1 axis played a prominent role in the regulation of GBM angiogenesis. Findings in this study will provide a new theory and experimental basis for GBM angiogenesis. More importantly, the MCM3AP-AS1/miR-211/KLF5/AGGF1 axis may serve as a new therapeutic target for the anti-angiogenic therapy of glioma.

## Author Contributions

YL contributed to the experiment design, implementation, manuscript draft, and data analysis. CY and JZ contributed to the experiment implementation and data analysis. YX conceived or designed the experiments. CY, HY, XL, and HC performed the experiments. JM, LL, ZL, and PW analyzed the data. CY conceived or designed the experiments, performed the experiments, and wrote the manuscript. All authors read and approved the final manuscript.

## Conflict of Interest Statement

The authors declare that the research was conducted in the absence of any commercial or financial relationships that could be construed as a potential conflict of interest.
